The article "Characteristics of Plantar Pressure Distribution in Diabetes with or without Diabetic Peripheral Neuropathy and Peripheral Arterial Disease" was published in 2022. Journal: J Healthc Eng.

# Characteristics of Plantar Pressure Distribution in Diabetes with or without Diabetic Peripheral Neuropathy and Peripheral Arterial Disease

**DOI:** 10.1155/2022/2437831

**Published:** 2022-06-06

**Authors:** Zijun Cao, Fang Wang, Xuemei Li, Jun Hu, Yaoguang He, Jianguo Zhang

**Affiliations:** ^1^College of Mechanical Engineering, Tianjin University of Science and Technology, Tianjin 300222, China; ^2^Key Laboratory of Integrated Design and Online Monitoring, Light Industry and Food Machinery and Equipment,Tianjin, Tianjin300222, China; ^3^Key Laboratory of Human Motion Analysis and Rehabilitation Technology of the Ministry of Civil Affairs, National Research Centre for Rehabilitation Technical Aids,No. 1 Ronghuazhonglu,BDA, Beijing 100176, China; ^4^NHC Key Laboratory of Hormones and Development, Tianjin Key Laboratory of Metabolic Diseases, Chu Hsien-I Memorial Hospital and Tianjin Endocrinology InstituteTianjin Medical University, Tianjin 300134, China

## Abstract

**Background:**

Excessive plantar pressure leads to increased risk of diabetic foot ulcers. Diabetic peripheral neuropathy (DPN) and peripheral arterial disease (PAD) have been considered to be associated with alterations in gait and plantar pressure in diabetic patients. However, few studies have differentiated the effects with each of them.

**Objective:**

To investigate the plantar pressure distribution in diabetic patients, with DPN and PAD as independent or combined factors.

**Methods:**

112 subjects were recruited: 24 diabetic patients with both DPN and PAD (DPN-PAD group), 12 diabetic patients with DPN without PAD (DPN group), 10 diabetic patients with PAD without DPN (PAD group), 23 diabetic patients without DPN or PAD, and 43 nondiabetic healthy controls (HC group). The in-shoe plantar pressure during natural walking was measured. Differences in peak pressure, contact area, proportion of high pressure area (%HP), and anterior/posterior position of centre of pressure (COP) were analysed.

**Results:**

Compared with HC group, in DPN-PAD group and DPN group, the peak pressures in all three forefoot regions increased significantly; in PAD group, the peak pressure in lateral forefoot increased significantly. The contact area of midfoot in the DPN-PAD group decreased significantly. PAD group had larger HP% of lateral forefoot, DPN group had larger HP% of inner forefoot, and DPN-PAD group had larger HP% of total plantar area. There was a significant tendency of the anterior displacement of COP in the DPN-PAD group and DPN group. No significant differences were observed between the D group and HC group.

**Conclusion:**

DPN or PAD could affect the plantar pressure distribution in diabetic patients independently or synergistically, resulting in increased forefoot pressure and the area at risk of ulcers. DPN has a more pronounced effect on peak pressure than PAD. The synergistic effect of them could significantly reduce the plantar contact area of midfoot.

The article "Characteristics of Plantar Pressure Distribution in Diabetes with or without Diabetic Peripheral Neuropathy and Peripheral Arterial Disease" was published in 2022. Journal: J Healthc Eng.

## 1. Introduction

Diabetic patients are prone to many complications during the course of disease. Diabetic foot syndrome is one of the most serious chronic complications of diabetes mellitus, leading to foot ulcers or even lower extremity amputation. Diabetic foot ulcer (DFU) is the most common cause of nontraumatic limb amputation [1]. It is estimated that the lifetime risk of a diabetic patient developing DFU could be as high as 30% [2], and the recurrence risk within 5 years after ulcer healing was 65% [3]. The treatment and prevention of DFU is a worldwide concern.

DFU is associated with multiple factors. The main pathophysiological factors include peripheral neuropathy, macroangiopathy, and the repetitive trauma caused by increased plantar pressure [4]. Other components include microangiopahy, callus, and foot deformity [5, 6]. The physical trauma heals relatively rapidly in healthy foot tissue under appropriate conditions. However, the healing process in diabetics is impaired, and the trauma is susceptible to infection and eventually ulcers.

Diabetic peripheral neuropathy (DPN) is a common complication in diabetic patients. DPN could lead to reduced peripheral sensation and compromised proprioceptive feedback control of human locomotion [7]. Motor neuropathy causes weakening muscle strength and altered gait. The loss of protective sensitivity leads to reduction in the perception of pain and increased plantar pressure [8]. Rahman et al. [9] reported a decreased in-shoe peak pressure during shod walking in rearfoot in diabetics with DPN compared to healthy people. Guldemond et al. [10] reported increased peak pressure in plantar forefoot region in diabetics with DPN compared to diabetics without DPN during barefoot walking. In Gnanasundaram et al.'s study [11], diabetics with or without DPN had higher peak pressure in medial heel region compared to healthy people, while no significant differences were found between diabetics with and without DPN. These studies have shown differences in pressure distribution between shod walking and barefoot walking. Owings et al. [12] suggested that in-shoe pressure was a more realistic variable than barefoot pressure for the screening and examination of foot ulceration risk in diabetic patients, considering that people wear shoes most of the time in daily activities.

Peripheral arterial disease (PAD) is a progressive disease caused by the atherosclerosis that leads to ischemia of lower limb tissue and promotes the development of ulcers [13]. There were 202 million PAD patients worldwide [14]. People with diabetes have four times the risk of PAD than people without diabetes [15], and two-thirds of chronic, nonhealing plantar ulcers have arterial insufficiency [16]. The presence of PAD and diabetes reduced mass and function via multiple mechanisms in synergistic way [17]. Altered spatiotemporal gait parameters, such as decreased step length, cadence, and velocity in patients with PAD, have been reported [18]. A typical symptom of PAD is intermittent claudication, characterized by the cramping pain in legs after short walks [19]. Szymczak et al. [20] suggested that PAD patients with and without intermittent claudication have shorter step length than healthy subjects. Cheung et al. [17] reported that patients with diabetes and PAD had significantly lower gait speed compared with subjects without diabetes or PAD, while no such difference was found in the diabetics without PAD and the PAD patients without diabetes. Pataky et al. [21] reported a significant correlation between plantar pressure under the first metatarsal head and Doppler arterial pressure of both tibial posterior and dorsalis pedis artery in diabetic patients with both peripheral neuropathy and vascular disease. Mantovani et al. [22] reported a higher pressure-time integral in diabetic patients with both peripheral neuropathy and peripheral vasculopathy compared with nondiabetic patients. They suggested that the gait pattern worsened with the severity of clinical impairment.

The article "Characteristics of Plantar Pressure Distribution in Diabetes with or without Diabetic Peripheral Neuropathy and Peripheral Arterial Disease" was published in 2022. Journal: J Healthc Eng.

Previous studies have mainly focused on the plantar pressure in diabetic patients with neuropathy rather than vasculopathy. Moreover, few studies have removed the influences of PAD in patients with DPN or removed the influence of DPN in patients with PAD. Thus, there was a gap in knowledge about how DPN and PAD affect plantar pressure in diabetic patients independently or synergistically. The aim of this study was to investigate the characteristics of in-shoe plantar pressure during natural walking in diabetic patients with DPN or PAD, more specifically, to assess the plantar pressure parameters in diabetic patients “with DPN and PAD,” “with DPN without PAD,” “with PAD without DPN,” and “without DPN or PAD.” Identifying the changes in plantar pressure could contribute to awareness of the risks of diabetic complications and help improve therapy interventions such as exercise programs or therapy footwear.

## 2. Materials and Methods

### 2.1. Participants

112 subjects were recruited in this study: 24 diabetics with DPN and PAD (DPN-PAD group), 12 diabetics with DPN and no PAD (DPN group), 10 diabetics with PAD and no DPN (PAD group), 23 diabetics without either DPN or PAD (D group), and 43 nondiabetic healthy controls (HC group). Patients were recruited from Tianjin Medical University Chu Hsien-I Memorial Hospital. The study was approved by the Institutional Review Board of Tianjin University of Science and Technology. All experiments were performed in accordance with the World Medical Association's Declaration of Helsinki. Subjects involved were informed of the research procedure and signed the informed consent. Demographic and anthropometric data of subjects are shown in Table 1.

The article "Characteristics of Plantar Pressure Distribution in Diabetes with or without Diabetic Peripheral Neuropathy and Peripheral Arterial Disease" was published in 2022. Journal: J Healthc Eng.

Data of age, height, weight, and BMI were obtained from medical records or by interview. The diagnosis of DPN and PAD and HbA1c levels were obtained from medical records of diabetes patients. Subjects were excluded if they had any of the followings: current or a history of foot ulcers, foot deformity, lower limb amputations in either limb, and unable to walk repeatedly unaided over a distance of 10 m. The presence of intermittent claudication was not considered in PAD patients. In this study, the plantar pressure data of subjects were collected for walking 10 meters, which was much shorter than the distance of the onset of intermittent claudication (usually a few hundred meters). In addition, several studies have revealed altered gait parameters in PAD patients both with and without intermittent claudication [23, 24].

### 2.2. Plantar Pressure Measurements and Statistical Analysis

The plantar pressure experiment was carried out with T&T Medilogic 5.8.1 measurement system (NORAXON, USA). The dynamic sampling frequency was 300 Hz. Uniform flat shoes and thin cotton socks with suitable sizes were assigned to subjects. All subjects walked 10 meters on a straight walkway with self-selected speed and stride length.

The plantar pressure in steady gait cycle was included for analysis, and data of initial and terminal stage were excluded to eliminate the effects of acceleration and deceleration. The plantar area was segmented into 7 regions, namely, toes, lateral forefoot, inner forefoot, medial forefoot, midfoot, lateral heel, and medial heel, respectively. The schematic image of plantar regions is shown in Figure 1. The absolute value and normalized (scale to body weight) value of peak pressure, normalized plantar contact area (scale to total plantar area), and the proportion of high pressure area (%HP) in segmented regions were calculated. High-pressure was defined as the absolute value above 200 kPa.

The trajectory of centre of pressure (COP) formed butterfly diagram. The anterior/posterior position of COP was the distance between the intersection point of butterfly diagram and the zero position (initial contact position), as shown in Figure 2. The value of each subject was normalized by the foot length, and the ratios of each group were calculated.

The article "Characteristics of Plantar Pressure Distribution in Diabetes with or without Diabetic Peripheral Neuropathy and Peripheral Arterial Disease" was published in 2022. Journal: J Healthc Eng.

Statistical analysis was performed using SPSS software 21.0 (IBM, USA). Mean and standard deviation of each group were calculated. Kolmogorov–Smirnov test was performed to assess normal distribution. One-way ANOVA was performed to analyse the differences of plantar pressures between the four diabetic groups and control group, and the significant level of the differences was 0.05.

## 3. Results

### 3.1. Absolute and Normalized Peak Pressure

The absolute peak pressures are shown in Table 2. In each group, the peak pressure in inner forefoot was higher than that in medial forefoot and lateral forefoot, and the peak pressure in lateral heel was higher than that in medial heel. The absolute peak pressures in all regions except midfoot were higher than 200 kPa.

The normalized peak pressures and the results of difference analysis between groups are shown in Table 3. Compared with the HC group, the normalized peak pressures in all three forefoot regions in the DPN-PAD group and DPN group were significantly higher, and the peak pressure in lateral forefoot in PAD was significantly higher. No significant differences were observed between D group and HC group.

### 3.2. Plantar Contact Area

The normalized plantar contact area is shown in Table 4. Compared with the HC group, the contact area of midfoot in the DPN-PAD group was significantly smaller. Although no significant differences were observed in other groups, there was a tendency of decreasing contact area of midfoot in the DPN group, PAD group and D group. In addition, the experimental peak pressure distribution during whole gait cycle of the subjects in different groups is shown in Figure 3. DPN-PAD group had the smallest contact area, especially in midfoot, which was consistent with the results in Table 4. Compared with the HC group, there was also a decreasing tendency of contact area of midfoot in the DPN group and PAD group, particularly in the PAD group.

### 3.3. Proportion of the High Pressure Area

The HP% of segmented plantar regions is shown in Table 5. Compared with the HC group, the HP% of total plantar area in the DPN-PAD group was significantly larger, while no significant differences were found in segmented regions. The significant increases were also observed in the inner forefoot in DPN group and lateral forefoot in PAD group. Though the differences of HP% of lateral forefoot in DPN-PAD group and DPN group were not significant compared with the HC group, there was still a tendency of increase. No significant differences were observed between the D group and HC group.

The article "Characteristics of Plantar Pressure Distribution in Diabetes with or without Diabetic Peripheral Neuropathy and Peripheral Arterial Disease" was published in 2022. Journal: J Healthc Eng.

### 3.4. Anterior/Posterior Position of COP

The normalized anterior/posterior position of COP is shown in Table 6. Compared with the HC group, a significant increase was observed in the DPN-PAD group and DPN group. No significant differences were found in the other groups.

## 4. Discussion

As shown in Table 3, DPN or PAD could independently lead to increased peak pressure in forefoot. Raspovic [25] reported reduced motion at the ankle, less foot rotation, and less fist metatarsophalangeal joint movement in subjects with peripheral neuropathy and a history of plantar ulceration. Gardner et al. [26] reported reduced swing phase and extended stance phase in PAD patients. These may lead to the accumulation of load in forefoot region as well as the increased plantar pressure. Significant increases of peak pressures were observed in all three forefoot regions in DPN group, while only in lateral forefoot in the PAD group. It seemed that DPN had a greater effect on peak pressure than PAD. Similar to the DPN group, the peak pressures in the three forefoot regions in DPN-PAD group were significantly increased, but the pressure value was close. The combination of neuropathy and arterial disease did not further increase the peak pressure.

Although the difference of peak pressure in inner forefoot in PAD group was not significant compared with HC group, it also showed increasing tendency and the pressure level was close to that of DPN-PAD group. This suggested that the alteration of plantar pressure in diabetic patients with PAD began in lateral forefoot, followed by inner forefoot. Atherosclerosis resulted in insufficient oxygen and nutrients. Long-term vasculopathy causes altered muscle morphology and mitochondrial function, resulting in decreased muscle strength [17]. Myers et al. [27] reported the alteration of joint kinematics and kinetics in patients with PAD during pain-free walking compared with healthy subjects. They found decreased dorsiflexor torque of ankle during stance phase in PAD patients. In addition, the kinematic changes of greater ankle plantarflexion angle reduced time to peak plantar flexion and increased time to peak dorsiflexion in patients with PAD resulted in altered foot rotation [28]. The alteration of plantar pressure in PAD group was accompanied by these changes of gait parameters.

To the author's knowledge, the plantar contact area during walking in these specific populations has not been reported. Pataky et al. [29] reported a significantly reduced contact area in diabetic patients without peripheral neuropathy or peripheral arterial disease compared to nondiabetic subjects. However, it was the contact area in static standing position they investigated. As shown in Table 4 and Figure 3, the contact area of midfoot in DPN-PAD patient and PAD patient was relatively small, which may reflect a reduction in plantar soft tissue. It has been reported that the presence of both diabetes and PAD could reduce muscle mass via multiple mechanisms synergistically [30, 31]. Long-term hyperglycemia and ischemia damage not only lower limb muscles but also plantar soft tissue. Thinner and stiffer soft tissue is also associated with increased plantar pressure [32]. PAD causes reduced supply of oxygen and nutrients, resulting in alteration in histological characters of plantar soft tissue. Ischemia promotes the plantar soft tissue thickness under 1st and 5th metatarsal heads reduction [29]. Thinner soft tissue could also contribute to higher plantar pressure. The elevated repetitive mechanical stress, in turn, increases the fragility of microvessel and decreases blood flow, producing a vicious cycle [23].

The article "Characteristics of Plantar Pressure Distribution in Diabetes with or without Diabetic Peripheral Neuropathy and Peripheral Arterial Disease" was published in 2022. Journal: J Healthc Eng.

In DPN group, no significant differences of segmented contact area were observed, but significant increase of peak pressures were observed in all three forefoot regions. This suggested that the increased peak pressure may not be due to the altered contact area, but to the tendency of the anterior displacement of weight-bearing, which was confirmed by the results in Table 5. Compared with the HC group, all four diabetic groups showed a tendency of the anterior displacement of COP, and the significant differences were observed in the DPN-PAD group and DPN group. Similar conclusion was also presented in previous research. Melai et al. [33] observed a faster forward transfer of centre of pressure and consequently higher load in forefoot in patients with DPN.

Another important parameter analysed in this study was the proportion of the high pressure area. Owings et al. [12] investigated the in-shoe plantar pressure in diabetic patients with DPN and a history of DFU and suggested 200 kPa as a reference in foot ulceration prevention. This value was obtained from the position of healed ulcers in diabetic patients with a history of ulcers and was considered safe for diabetic with or without a history of ulcers. It has been widely used in later studies as a threshold for classifying high pressure or as and optimization target for developing offloading footwear [34–36]. As shown in Table 5, the HP% of the lateral forefoot in PAD group and the inner forefoot in DPN group was significantly larger than that in the HC group. Although there were no significant differences of segmented HP% between the DPN-PAD and HC group, the HP% of total plantar area was significantly higher. Moreover, a tendency of increasing HP% was also observed in all lateral forefoot and inner forefoot regions in DPN-PAD, DPN, and PAD groups compared with the HC group, although the differences were not significant. The HP% is positively associated with peak pressure in segmented plantar regions. Either peripheral neuropathy or peripheral arterial disease could independently cause increased plantar pressure and high pressure area. The combination of neuropathy and vasculopathy did not cause further increases of peak pressure, but caused larger area of high pressure.

The article "Characteristics of Plantar Pressure Distribution in Diabetes with or without Diabetic Peripheral Neuropathy and Peripheral Arterial Disease" was published in 2022. Journal: J Healthc Eng.

A noteworthy result in our study is that compared with the HC group, no significant differences of plantar pressure parameters were observed in the D group. The consistent results have been found in other study [11]. However, there was a tendency of decreasing of contact area in the D group, as shown in Table 4. This may indicate that the alteration of soft tissue character occurred in the diabetic stage before the presence of complications. The progressive effects of changes in peripheral nervous system and vessels on the lower limb physiology making the changes in plantar pressure was a gradual process. The significant changes in plantar pressure occurred after the combination of DPN or PAD.

However, the lack of significant differences between the D group and HC group differs from Pataky's [29]. They found significant differences of peak pressure under the big toe, 5th metatarsal head, and heel in diabetic patients without peripheral neuropathy or vasculopathy compared with nondiabetic subjects. In this study, the absolute values of peak pressure in all three forefoot regions in the D group showed a tendency to increase, but the normalized values did not. The inconsistent results suggested that the body weight of subjects should be a concern. Although an appropriate range of body weight and BMI have been adopted as one of the inclusion criteria in many studies, the differences of body weight in individuals still affected plantar pressure. In the study of Castro et al. [37, 38], the results of analysing absolute value of ground reaction force and plantar pressure were different from the results of analysing normalized value of ground reaction force and plantar pressure. Therefore, the absolute value could be used to indicate the magnitude of plantar pressure and evaluating the risk of ulceration, while the normalized value should be used in analysis of differences between groups to subtract the effects of body weight.

A potential limitation of this study is that the microvascular complications such as nephropathy and retinopathy was not considered. Future research on potential factors associated with macroangiopathy and microangiopathy could be helpful to further understand the mechanism of the plantar pressure alteration in diabetic patients. The current results could be considered as a preliminary demonstration of the independent and synergistic effects of DPN and PAD on plantar pressure in diabetic patients.

The article "Characteristics of Plantar Pressure Distribution in Diabetes with or without Diabetic Peripheral Neuropathy and Peripheral Arterial Disease" was published in 2022. Journal: J Healthc Eng.

## 5. Conclusions

The current study provides the evidence for learning the independent or synergistic effects of peripheral neuropathy and peripheral arterial disease on plantar pressure in diabetic patients. Identifying the changes in plantar pressure distribution helps to carry out physical therapy interventions, such as exercise program, offloading footwear, and therapeutic orthosis. The alteration of plantar pressure in diabetic patients was a gradual process, and significant changes occurred after the combination of DPN or PAD. DPN and PAD could independently affect plantar pressure in diabetic patients, leading to higher pressure in forefoot and larger area at risk of ulcers. The prevention and/or control of DPN and PAD and the redistribution of plantar pressure from forefoot onto the whole foot should be highlighted in clinical practice.

## Figures and Tables

**Figure 1:** Segmented plantar regions.

**Figure 2:** Anterior/posterior position of COP.

**Figure 3:** Peak plantar pressure distribution during the gait cycle.

**Table 1:** Demographic and anthropometric data of subjects.

Variables	DPN-PAD	DPN	PAD	D	HC
Number (M/F)	24 (13/11)	12 (6/6)	10 (7/3)	23 (16/7)	43 (23/20)
Age (years)	60.4 ± 7.6	55.0 ± 13.3	55.8 ± 15.0	54.4 ± 12.1	57.6 ± 15.4
Height (cm)	165.9 ± 8.6	166.5 ± 4.4	167.8 ± 6.7	168.2 ± 9.0	166.5 ± 6.9
Weight (kg)	68.4 ± 7.2	66.6 ± 12.8	76.4 ± 5.2	73.1 ± 11.1	67.1 ± 8.3
BMI (kg/m^2^)	24.9 ± 2.4	24.0 ± 4.2	27.2 ± 1.8	25.7 ± 2.5	24.2 ± 2.4
HbA1c (%)	8.6 ± 1.9	8.8 ± 1.7	8.4 ± 1.3	8.4 ± 1.9	—

**Table 2:** Absolute value of peak pressures in segmented plantar regions.

Region	DPN-PAD	DPN	PAD	D	HC
T	312.3 ± 141.3	264.3 ± 70.1	340.1 ± 64.6	294.4 ± 105.7	281.9 ± 106.7
LF	310.1 ± 120.1	325.6 ± 135.3	342.1 ± 114.3	262.9 ± 113.0	253.3 ± 90.8
IF	468.2 ± 121.2	524.1 ± 60.5	500.2 ± 128.4	422.6 ± 140.8	405.2 ± 120.3
MF	378.3 ± 109.9	372.7 ± 115.6	377.3 ± 125.6	341.9 ± 147.2	309.0 ± 102.1
M	143.6 ± 88.9	173.4 ± 104.8	129.7 ± 51.8	135.7 ± 74.4	155.0 ± 96.7
LH	456.1 ± 105.4	417.8 ± 93.1	454.3 ± 84.5	415.8 ± 124.8	422.2 ± 100.5
MH	439.5 ± 100.3	385.6 ± 87.7	422.9 ± 75.6	407.8 ± 123.7	410.5 ± 102.2

The unit of peak pressure was kPa. Abbreviations: T = toes; LF = lateral forefoot; IF = inner forefoot; MF = medial forefoot; M = midfoot; LH = lateral heel; MH = medial heel.

The article "Characteristics of Plantar Pressure Distribution in Diabetes with or without Diabetic Peripheral Neuropathy and Peripheral Arterial Disease" was published in 2022. Journal: J Healthc Eng.

**Table 3:** Normalized (scale to body weight) value of peak pressures in segmented plantar regions.

Region	Normalized peak pressure					*P* value			
	DPN-PAD	DPN	PAD	D	HC	DPN-PAD vs. HC	DPN vs. HC	PAD vs. HC	D vs. HC
T	4.6 ± 2.1	4.1 ± 1.0	4.5 ± 0.9	4.0 ± 1.2	4.3 ± 1.7	0.514	0.633	0.701	0.483
LF	4.6 ± 1.8^*∗*^	4.7 ± 2.3^*∗*^	4.5 ± 1.5^*∗*^	3.6 ± 1.5	3.7 ± 1.2	0.035^*∗*^	0.039^*∗*^	0.045^*∗*^	0.688
IF	6.9 ± 1.7^*∗*^	7.6 ± 2.0^*∗*^	6.6 ± 1.7	5.8 ± 1.8	6.0 ± 1.4	0.043^*∗*^	0.021^*∗*^	0.320	0.597
MF	5.6 ± 1.4^*∗*^	5.8 ± 1.9^*∗*^	4.9 ± 1.8	4.6 ± 1.6	4.6 ± 1.3	0.010^*∗*^	0.019^*∗*^	0.556	0.975
M	2.1 ± 1.3	2.6 ± 1.5	1.7 ± 0.6	1.9 ± 1.0	2.3 ± 1.4	0.597	0.589	0.198	0.194
LH	6.7 ± 1.7	6.6 ± 2.0	6.0 ± 1.0	5.8 ± 1.8	6.4 ± 1.6	0.371	0.708	0.464	0.191
MH	6.5 ± 1.5	5.9 ± 1.3	5.5 ± 0.8	5.5 ± 1.3	6.1 ± 1.3	0.371	0.662	0.189	0.108

The unit of peak pressure was kPa; the unit of body weight was kg. Values with^*∗*^ indicate statistically significant difference(*P* < 0.05) compared with HC group. T = toes; LF = lateral forefoot; IF = inner forefoot; MF = medial forefoot; M = midfoot; LH = lateral heel; MH = medial heel.

**Table 4:** Normalized value (scale to total plantar contact area) of contact area of segmented plantar regions.

Region	Normalized contact area (%)					*P* value			
	DPN-PAD	DPN	PAD	D	HC	DPN-PAD vs. HC	DPN vs. HC	PAD vs. HC	D vs. HC
T	17.5 ± 1.4	17.1 ± 1.9	16.8 ± 1.4	16.9 ± 2.1	17.4 ± 1.8	0.94	0.617	0.330	0.267
LF	7.0 ± 0.8	6.9 ± 1.1	6.8 ± 1.1	7.2 ± 1.1	7.0 ± 2.0	0.907	0.867	0.679	0.710
IF	9.8 ± 0.8	9.6 ± 0.6	9.5 ± 0.8	9.6 ± 0.7	9.6 ± 1.6	0.562	0.946	0.905	0.872
MF	9.0 ± 1.5	9.2 ± 1.5	9.3 ± 1.0	9.0 ± 1.2	8.7 ± 2.2	0.601	0.482	0.464	0.554
M	25.8 ± 4.1 ^*∗*^	26.7 ± 3.5	26.2 ± 3.8	26.8 ± 3.6	29.3 ± 4.9	0.005^*∗*^	0.101	0.217	0.097
LH	16.4 ± 2.3	16.6 ± 2.1	16.8 ± 1.5	16.4 ± 2.0	16.0 ± 3.4	0.555	0.529	0.459	0.573
MH	14.5 ± 1.2	13.7 ± 1.5	13.6 ± 1.6	14.1 ± 1.3	14.4 ± 2.7	0.883	0.382	0.363	0.581

Values with ^*∗*^ indicate statistically significant difference (*P* < 0.05) compared with HC. Abbreviations T = toes; LF = lateral forefoot; IF = inner forefoot; MF = medial forefoot; M = midfoot; LH = lateral heel; MH = medial heel; total = total plantar area.

**Table 5:** HP% of segmented and total plantar regions.

Region	HP% (%)					*P* value			
	DPN-PAD	DPN	PAD	D	HC	DPN-PAD vs. HC	DPN vs. HC	PAD vs. HC	D vs. HC
T	13.1 ± 12.2	11.3 ± 7.5	16.2 ± 7.0	15.6 ± 11.7	11.6 ± 9.0	0.581	0.901	0.146	0.132
LF	28.1 ± 18.4	30.5 ± 20.7	32.1 ± 17.7^∗^	22.6 ± 22.0	20.0 ± 16.6	0.075	0.063	0.049^∗^	0.603
IF	55.6 ± 18.6	66.9 ± 15.1^∗^	59.5 ± 11.7	45.4 ± 19.7	51.8 ± 22.2	0.485	0.033^∗^	0.319	0.260
MF	32.5 ± 18.4	27.2 ± 15.1	22.4 ± 10.5	26.3 ± 18.5	26.0 ± 17.4	0.166	0.838	0.531	0.963
M	2.0 ± 4.0	2.3 ± 3.2	0.6 ± 1.0	1.1 ± 2.1	1.5 ± 3.0	0.637	0.440	0.338	0.517
LH	41.9 ± 13.5	36.6 ± 10.4	42.6 ± 12.5	36.8 ± 17.4	39.0 ± 14.5	0.427	0.607	0.482	0.595
MH	34.9 ± 11.0	31.2 ± 9.7	34.3 ± 8.9	33.9 ± 14.5	32.1 (10.0)	0.298	0.797	0.530	0.556
Total	25.1 (7.1)^∗^	24.0 (3.9)	24.7 (5.0)	22.1 (8.7)	21.4 (6.4)	0.035^∗^	0.204	0.147	0.729

Values with ^∗^indicate statistically significant difference (*P* < 0.05) compared with HC. Abbreviations: HP% = proportion of high pressure (>200 kPa) area; T = toes; LF = lateral forefoot; IF = inner forefoot; MF = medial forefoot; M = midfoot; LH = lateral heel; MH = medial heel. Total is the proportion of high pressure area in the total plantar area.

The article "Characteristics of Plantar Pressure Distribution in Diabetes with or without Diabetic Peripheral Neuropathy and Peripheral Arterial Disease" was published in 2022. Journal: J Healthc Eng.

**Table 6:** Anterior/posterior position of COP in each group.

Anterior/posterior position of COP (%)					*P* value			
DPN-PAD	DPN	PAD	D	HC	DPN-PAD vs. HC	DPN vs. HC	PAD vs. HC	D vs. HC
55.0 ± 2.6^∗^	54.6 ± 1.9^∗^	52.7 ± 4.4	52.4 ± 3.2	51.4 ± 3.0	0.001^∗^	0.002^∗^	0.285	0.224

Values with ^∗^indicate statistically significant difference (*P* < 0.05) compared with HC. Abbreviations: T = toes; LF = lateral forefoot; IF = inner forefoot; MF = medial forefoot; M = midfoot; LH = lateral heel; MH = medial heel; total = total plantar area.

## Data Availability

The raw/processed data required to reproduce these findings cannot be shared at this time as the data also form part of an ongoing study.
